# Mastering uncertainty: A predictive processing account of enjoying uncertain success in video game play

**DOI:** 10.3389/fpsyg.2022.924953

**Published:** 2022-07-26

**Authors:** Sebastian Deterding, Marc Malmdorf Andersen, Julian Kiverstein, Mark Miller

**Affiliations:** ^1^Dyson School of Design Engineering, Imperial College London, London, United Kingdom; ^2^Digital Creativity Labs, University of York, York, United Kingdom; ^3^Interacting Minds Centre, School of Culture and Society, Aarhus University, Aarhus, Denmark; ^4^Department of Psychiatry, Amsterdam University Medical Centre, Amsterdam, Netherlands; ^5^Centre for Consciousness and Contemplative Studies, Monash University, Melbourne, VIC, Australia; ^6^Center for Human Nature, Artificial Intelligence and Neuroscience, Hokkaido University, Sapporo, Japan

**Keywords:** active inference, predictive processing, video games, game enjoyment, gaming motivation, uncertainty, competence

## Abstract

Why do we seek out and enjoy uncertain success in playing games? Game designers and researchers suggest that games whose challenges match player skills afford engaging experiences of achievement, competence, or effectance—of *doing well*. Yet, current models struggle to explain why such balanced challenges best afford these experiences and do not straightforwardly account for the appeal of high- and low-challenge game genres like Idle and Soulslike games. In this article, we show that Predictive Processing (PP) provides a coherent formal cognitive framework which can explain the fun in tackling game challenges with uncertain success as the dynamic process of reducing uncertainty surprisingly efficiently. In gameplay as elsewhere, people enjoy *doing better than expected*, which can track learning progress. In different forms, balanced, Idle, and Soulslike games alike afford regular accelerations of uncertainty reduction. We argue that this model also aligns with a popular practitioner model, Raph Koster’s *Theory of Fun for Game Design*, and can unify currently differentially modelled gameplay motives around competence and curiosity.

## Introduction

While much of modern, bureaucratised society is geared toward *reducing* uncertainty, games are strange pockets of social life designed to *heighten* it—much to the attraction of players and spectators entering these pockets (Malaby, 2003; Costykian, 2013). This crucially includes *uncertain success*. Several scholars like Caillois (2001, p. 7) went so far as to *define* games and play as ‘uncertain activity. Doubt must remain until the end…. An outcome known in advance, with no possibility of error or surprise, … is incompatible with the nature of play’ (see also Malaby, 2007; Bateman, 2011; Costykian, 2013). This view is also common among contemporary game designers. To quote Elias et al. (2012, p. 137): ‘if we had to pick one ingredient that was necessary… for something to be a game, uncertainty in outcome would probably be it.’

Games afford uncertain outcomes through a variety of ways, such as the randomness of a dice roll or the hidden information of the opponent’s Poker hand. One important way, particularly in games of skill, is some form of balanced or *optimal challenge*: here, uncertainty over the player overcoming an obstacle or other player is first maximized by matching players with opponents or obstacles of equal strength, and then resolved, one way or another (Elias et al., 2012, p. 137–166; Costykian, 2013).

One key question for games research is *why* people seek out and enjoy uncertain success.^1^ While current theories see gameplay fuelled by multiple motives (e.g., Vanden Abeele et al., 2020; Klimmt and Possler, 2021), they typically explain the appeal of optimal challenge with intrinsic motivations of achievement, competence, or effectance (‘ACE’ henceforth). Broadly, ACE theories hold that people need and therefore seek out the positively valenced experience of effectively causing intended change in the world: We enjoy succeeding or *doing well* at something (Klimmt and Possler, 2021). Yet if gameplay is motivated by enjoying success, why would we seek *un-*certain success? As we will show, among ACE theories, only achievement theory offers a robust answer. But even this explanation is troubled by two recent popular game genres that sit on either end of the challenge spectrum: Idle games with no apparent challenge (Alharthi et al., 2018), and Soulslike games that promise long sequences of failure even for skilled players (Petralito et al., 2017).

In this theoretical paper, we propose that the neurocognitive and neurocomputational framework of predictive processing (PP; Clark, 2015; Parr et al., 2022) provides a coherent account of why we seek and enjoy uncertain success that can explain optimal challenge, Idle games, and Soulslike games alike. We first set out current research on the appeal of uncertain success in games, how ACE theories account for it, and where they fall short. We then give a brief introduction into PP, which has seen a rapid ascent in the cognitive sciences, but also more recently in play research and neuroaesthetics (Frascarolli et al., 2021; Andersen et al., 2022). PP sees living beings as aiming to minimise *prediction error* – that is, mismatches between predicted and actual states. In this account, uncertainty is parsed as *expected* prediction error (Friston et al., 2017). Colloquially, the more uncertain we are about a belief about what will happen next, the likelier we think that this belief will be proven erroneous. Living beings orient themselves toward actions that promise the fastest reduction of expected prediction error. Momentary jolts of positive affect emerge whenever uncertainty is reduced *faster than expected* (Kiverstein et al., 2019). This core mechanism of PP, we will demonstrate, can elegantly explain the appeal of optimal challenges in games, but also of Idle and Soulslike games. And it provides a neurocognitive account that is largely compatible with a highly influential practitioner model, Koster’s (2005) *Theory of Fun for Game Design*.

Our discussion contextualises PP within other (neuro) computational models of intrinsic motivation and teases out characteristics and contributions in the context of games research and practice: PP provides precise formalizations that lend themselves to experimental testing, new research paradigms, and practical applications. It accounts for emerging empirical work on the importance of expectations in game engagement. Finally, by showing how PP can explain why people seek out and enjoy optimal challenge, we hope to pave the way for a unifying framework that can also account for the appeals of novel content, narrative suspense, and other forms of uncertainty in games.

## Uncertain success in games

Different research communities have framed uncertainty in games in different ways. The *game design* literature chiefly unpacks different person-external, material sources of uncertainty (Elias et al., 2012; Costykian, 2013), which are differently prevalent in different types or genres of games. For instance, games of chance (or *alea*, Caillois, 2001, p. 17–19) may feature material randomness generators like dice, card decks, or Roulette wheels. We will refer to this as *external uncertainty*. External uncertainty is often information-theoretically modelled and quantified as probability distributions over alternative possible game states or outcomes given some observed information, resulting in uncertainty measures like Shannon entropy (Klir, 2006). This quantification can also comprise the (real or expected) precision and accuracy of the information we use to predict outcomes. As different actors can have different information states (especially in games with imperfect and/or asymmetrical information, like Poker), one can model ‘subjective’ uncertainty from an individual actor’s information state.

This is not to be confused with uncertainty as a person-internal, conscious subjective experience, which we will call *felt uncertainty*. Studying this lived experience has been the main thrust in *player research*, resulting in self-report instruments capturing common sources of felt uncertainty in play (Power et al., 2019), or taxonomies of motivating, positively valenced uncertainty (Kumari et al., 2019).

This differs yet again from *cognitive science, psychology, and behavioural economics* studying perception, action, and decision-making under uncertainty: how people choose to sample new information or act when they do not know with certainty the state of the world, or which option is optimal for them (Crupi et al., 2018). Work in this vein again usually uses information-theoretical formalisations to model how cognitive systems compute and work to reduce and resolve the uncertainty of their beliefs and decisions. We will refer to this as *cognitive uncertainty*. Cognitive uncertainty is taken to occur chiefly sub-personally or unconsciously, although sub-personally computed cognitive uncertainty can give rise to felt uncertainty and is often afforded by external uncertainty. PP squarely falls into the cognitive camp: It argues that our cognitive systems, implemented in the human brain, operate by constructing, weighing, and testing alternative hypotheses about the world against sensory data, aiming to continually reduce cognitive uncertainty, increasing its grip on the world.

In this article, we focus on the motivational appeal and positive experience of *one* form of external uncertainty in games: so-called outcome uncertainty over the success of a player afforded by optimal challenges. Importantly, outcome here not only refers to the end point of a game or match – as Costykian (2013, p. 10-11) observes, there are many games without clear end points. Rather, outcome refers to success relative to some goal a player set for themselves. Outcome uncertainty can thus occur and be resolved numerous times at many different time scales during one game session, from triggering a new attack combo to clearing a room of monsters to completing a campaign.

It is almost an axiom of contemporary games research and practice that well-designed games present *optimal challenges* that are neither trivially easy nor impossibly hard relative to the player’s current capabilities – statistically speaking, challenges that maximise outcome uncertainty. This notion of optimal challenge can be linked back to one of the earliest models in modern psychology, the Wundt Curve (Berlyne, 1970). Wundt observed an inverted-U relation between stimulus intensity and experience, where ‘optimal’ experience is found at a Goldilocks mid-point. Numerous early intrinsic motivation studies similarly observed such inverted-U curves, where maximal interest, positive affect, arousal, exploratory behavior, or behavioral persistence would show with medium levels of information incongruence, uncertainty, complexity, novelty, arousal, or task difficulty (for a review, see Deci, 1975).

In games research, as well as in the wider psychological literature, this idea of optimal challenge has arguably been most popularized by Csikszentmihalyi (1991). His flow theory proposes that a key phenomenological characteristic and antecedent of flow or ‘optimal experience’ is ‘when the challenges are just balanced with the person’s capacity to act’ (Csikszentmihalyi, 1991, p. 52). He later specified that ‘experiences that one believes are in the neighborhood of a 50/50 balance [of challenges and skills] are experienced as enjoyable’ (Csikszentmihalyi and Nakamura, 2010, p. 187), experimentally operationalized as, e.g., playing against a Chess opponent with an equal Elo Chess rating, or game outcomes close to a draw (Abuhamdeh and Csikszentmihalyi, 2012; Abuhamdeh et al., 2015). Today, the notion of optimal challenge (including a reference to flow) is found in most major game design textbooks (e.g., Schell, 2008; Fullerton, 2014; Macklin and Sharp, 2016), and central to the game design practices of balancing (Schreiber and Romero, 2021) and matchmaking (Graepel and Herbrich, 2006): presenting players with obstacles and opponents that are neither too hard, nor too easy. The paramount opinion among game designers is that a maximally fair and engaging match is one with equal (50:50) winning odds for each party. In single-player games, this has been translated into the assumption that an optimally balanced game features 50% winning odds for players (Lomas et al., 2017).

### Achievement, competence, and effectance theories

Assuming that games afford motivation and enjoyment through optimal challenges, this raises the obvious question: why? Why do people seek out, persist engagement in, and enjoy pursuing goals where their winning odds are below 100%? While most contemporary models assume that games afford multiple distinct motivating experiences in parallel (e.g., Vanden Abeele et al., 2020; Klimmt and Possler, 2021), the vast majority include and often centre on some notion of *achievement, competence,* or *effectance* (ACE). They agree that in tackling and overcoming the obstacles games pose, players feel a sense of effectively exercising their own capacities. This experience of *doing well* at a task is what is inherently enjoyable and motivating about gameplay (e.g., Klimmt, 2006; Rigby and Ryan, 2011; Zusho et al., 2014). Yet, on closer inspection, several current ACE theories lack satisfying accounts of *why* players would seek out optimal challenges.

#### Effectance

In a key article and follow-on monograph, White (1959, 1961) introduced the concept of *effectance* and broader competence theories to psychology. White held that play and similar exploratory behaviour could not be explained by then-dominant drive reduction theories. Rather, such activity is fuelled by ‘fun–because there is something inherently satisfying about it’ (White, 1961, p. 34). This inherent satisfaction is ‘a *feeling of efficacy* … of doing something, of being active or effective, of having an influence on something’ (*ibid*, p. 35). In everyday adult life, effectance experiences most commonly manifest in goal-directed action such as gameplay, ‘where we act with intentions to produce particular effects’ (*ibid.*, p. 35). In exploratory play, effectance arises not from attaining goals, but the sheer observation of the effects we produce in prodding the world. Effectance-seeking motivates exploratory behaviour resulting in learning – the build-up of *competence*, which White defined as ‘a person’s existing capacity to interact effectively with his environment’ (*ibid.*, p. 39).

In games research, Klimmt (2006) and Klimmt and Possler (2021) have most forcefully argued for effectance as a distinct gameplay motive and experience. For Klimmt, games generate effectance experiences on the level of moment-to-moment input–output loops between player and game. In good games, players receive immediate exaggerated feedback on every input—also known as ‘juicy’ feedback (Hicks et al., 2018): pressing the primary attack button in Hades (Standard Edition) (2018) reliably triggers a splashy audiovisual attack animation, for instance. This moment-to-moment effectance experience, Klimmt holds, is separate from that of competence, which for him is an experience that manifests on the higher organisational level of episode-by-episode pursuit of game goals. Thus, we can experience effectance without competence: in *Hades*, we may fail at our goal to kill all the monsters that spawned in a room and die, thwarting competence, and yet in the process, we enjoy the sheer agency experience of every button press reliably producing effects in the game world.

Now how does effectance motivation explain the appeal of uncertain success in games? Following Klimmt (2006), it does not: the attraction of uncertain success is about competence not effectance. White (1959, 1961) does not directly engage with uncertain success, but we can infer an answer from his observation that ‘effectance motivation subsides when a situation has been explored to the point that it no longer presents new possibilities’ (White, 1959, p. 322). In the action-feedback loop, there must be some *novel*, not yet learned ‘difference-in-sameness’ (*ibid.*). Thus, if a player were to replay *Hades* with the same weapon and primary attack over and over, increasingly discovering all their possible combinatorial results with different enemies, effectance experience would wane as there is less and less *novel* effectance. The player would therefore drift to explore other weapons, attacks, and possibly, other games which hold more–novel–effectance. As these are less well-learned, the player will also be less likely to succeed in their execution. Thus, players do not *directly* steer toward and enjoy uncertain success; rather, this is a side effect of their novelty-seeking. To explain why people do not get ‘stuck’ on a reliable source of effectance experience (or certain success) – happily sitting in a corner popping bubble wrap forever—White’s effectance motivation brings in some additional heterostatic conception of novelty-seeking or curiosity.^2^ This dynamic conception, as we will see, sits at the core of PP.

#### Competence

Whereas White sees competence as the learned capacities that result incidentally from effectance-motivated exploration, self-determination theory (SDT) considers effectance a subcomponent of a wider competence motive (Ryan and Deci, 2017). By some counts, SDT is presently the most frequently-used theory in empirical research on game enjoyment (Mekler et al., 2014; Tyack and Mekler, 2020), and widely used in the games industry (Rigby and Ryan, 2011). SDT posits that just like innate physiological needs such as hunger or thirst, humans have innate psychological needs that they need to satisfy to flourish, namely competence, autonomy, and relatedness. Intrinsically motivated action is energised and directed by the experiential enjoyment generated from satisfying these basic needs (Ryan and Deci, 2017, p. 117). We seek out, enjoy, and engage in video game play because it makes us feel competent, autonomous, and related (Ryan et al., 2006).

From the outset, SDT almost equates intrinsic motivation, especially competence satisfaction, with seeking-and-overcoming optimal challenges: ‘the needs for competence and self-determination keep people involved in ongoing cycles of seeking and conquering optimal challenges’ (Deci and Ryan, 1985, p. 33). Competence in SDT is defined as ‘feeling effective in one’s interactions with the social environment, that is, experiencing opportunities and support for the exercise, expansion, and expression of one’s capacities and talents’ (Ryan and Deci, 2017, p. 86).^3^

So what are optimal challenges in SDT, and why would competence satisfaction motivate us to tackle them? SDT argues that ‘intrinsic motivation is a *growth* function’ and therefore ‘manifested in circumstances in which people have the opportunity to exercise and stretch existing capacities or skills’, and not in circumstances ‘in which people have well mastered a skill… that would yield high rates of success but would not typically provide opportunities for growth’ (Ryan and Deci, 2017, p. 152). On the other hand, optimal challenge means ‘being regularly in a zone of mastery’ (*ibid.*, p. 153), because competence satisfaction is seen to arise from positive competence feedback: experiencing that one *is* good at a task, that one *does* succeed. SDT thus positions optimal challenge between certain, uncertain, and unlikely success: ‘Within SDT, then, optimal challenge means facing demands that most often one can master, rather than ones that are continuously at the leading edge of one’s capabilities. That type of high difficulty challenge should, however, be an intermittent element, in which case it can enhance and heighten intrinsic motivation’ (*ibid.*, p. 153).

Thus, SDT suggests that moderately difficult challenges (with at least *some* though not *maximally* uncertain success) are optimal for growth *and* intrinsic motivation, especially for competence satisfaction. And indeed, SDT authors argue that well-designed video games satisfy our competence need with optimal challenges, clear goals, and rich and varied positive competence feedback (Rigby and Ryan, 2011, p. 15–37). Several empirical studies have probed the impact of optimal challenge on competence experiences and intrinsic motivation in games, often with dynamic difficulty adjustment systems that are supposed to deliver optimal challenge (Keller and Bless, 2008; Klarkowski et al., 2016; Zohaib, 2018).

Yet on a closer look, this leaves open the question why challenges with *un*certain success (or a mixture of certain, uncertain, and unlikely success) would be most competence-need satisfying. If we enjoy and are motivated by feeling competent at a task thanks to positive competence feedback, tasks with the highest rate or likelihood of success (and thus, positive competence feedback) should be the most motivating, not tasks where we are likely to receive positive *and* negative competence feedback from time to time. Indeed, Ryan and Deci (2017, p. 156) lament the lack of studies examining or showing that tasks with moderate amounts of negative success feedback are motivating, let alone *more* motivating than those with only positive feedback:

“We have emphasized that intrinsic motivation is facilitated by optimally challenging activities, ones for which people could expect to fail some of the time and succeed some of the time. This implies that a modest amount of negative feedback […] may actually serve to challenge and thus motivate, rather than demotivate. Yet to date there is relatively little evidence for anything other than a perceived competence effect—namely, positive feedback that enhances perceived competence enhances intrinsic motivation, and negative feedback that diminishes perceived competence decreases intrinsic motivation.”

Put differently, the current SDT account of optimal challenge is internally incoherent: It acknowledges that seeking challenges with moderate to high difficulty (and therefore uncertain success) is optimal for competency growth—*getting better*—and therefore *should* be most intrinsically motivating and preferred. Yet that does not track with the logic that competence need satisfaction is constituted by experiences of *doing well*, which would be maximized by engaging tasks with certain success. Tasks with moderate difficulty can still instill competence experiences (upon success). But given free choice, competence-*maximising* agents should prefer tasks with certain over tasks with uncertain success.

This incoherence can be solved in at least two ways: One is that intrinsic motivation is fuelled not (just) by competence or *doing well*, but (also) by learning progress or *getting better*. As we will see, this is the solution PP proposes. A second solution is presented by achievement motivation theory: tasks of different difficulty present different informational signals about one’s competencies.

#### Achievement

The word ‘achievement’ looms large in game discourse: many games and game platforms feature so-called achievement systems—meta-game systems of optional goals whose attainment is tracked, displayed, and rewarded with a lasting signifier like a badge (Hamari and Eranti, 2011). ‘Achiever’ is one of four player types in an early influential typology of multi-user dungeon players. It designates players who preferentially enjoy acting on the game world and achieving in-game goals (Bartle, 1996).

In games design and research, achievement is often more or less equated with competence (e.g., Ryan et al., 2006; Vandenberghe, 2016). In psychology, in contrast, *achievement* marks a distinct construct and research tradition. For achievement motivation theory, achievement denotes ‘success in competition with a standard of excellence’ (McClelland et al., 1953, quoted in Reeve, 2015, p. 190). Following this theory, humans internalise how others evaluate them and turn these evaluations into social emotions of pride and shame. Succeeding at a standard of excellence—like jumping a certain length in sports—demonstrates socially desirable capacities and thus triggers positive emotions of pride, while failure evokes negative emotions of shame. People are both driven by a hopeful motive to approach success (and feel pride) and a fearful motive to avoid failure (and feel shame).

In Atkinson’s formal achievement motivation model (*ibid.*, p. 192–194), a person’s overall motivation to approach a standard of excellence (their Tendency to Succeed, *Ts*) comprises their Motivation to Succeed (*Ms*), the Probability of Success (*Ps*), and the Incentive Value of Success (*Is*): *Ts = Ms × Ps × Is*. Importantly, Atkinson models the Incentive Value as the direct inverse of the Probability of Success (*Is = 1*–*Ps*): the higher the bar, the more desirable competency is required and displayed when taking it. The mathematical upshot of this is a formal prediction of optimal challenge, in games and elsewhere: people will experience the strongest achievement motivation with tasks that have a 50% chance to succeed, as they create the largest product of success expectancy times signal value of success. If *Ps* = 0.5, then *Is* = 1*–Ps* = 0.5, and *Ts* = 0.5 *×* 0.5 = 0.25. Compare this to easy tasks (e.g., *Ps* = 0.9, *Is* = 0.1, *Ts* = 0.9 × 0.1 = 0.09) or hard tasks (*Ps* = 0.1, *Is* = 0.9, *Ts* = 0.1 × 0.9 = 0.09).^4^

Despite the wide currency of ‘achievement’ in game discourse, achievement motivation theory has found little adoption in research and practice (Zusho et al., 2014). To our knowledge, the only notable application to-date comes from Merrick (2016), who implemented formal models of achievement, power, and affiliation in AI game agents, with a view to affording more believable and diverse non-player character (NPC) behaviour. We cover achievement motivation theory here chiefly because among ACE theories, it provides the clearest and strongest (if not only) formal explanation for the motivational appeal of uncertain success.

### The puzzles of idle and soulslike games

In recent years, designers, critics, and scholars have taken increasing issue with the idea that games should, or do, exclusively centre on the pleasure of tackling and overcoming optimal challenges (e.g., Bateman, 2015; Paul, 2018). But even if we concede that tackling optimal challenges is but one of the many enjoyable experiences of gameplay, the last years have also seen the rise of two game genres at opposite ends of the challenge spectrum that put the very idea of optimal challenge into question: Idle and Soulslike games.

In so-called ‘Idle’ (or ‘Clicker’) games, there is no identifiable challenge: success and continuing progress are guaranteed, even in the absence of player action (Alharthi et al., 2018). These games [like Cookie Clicker (Standard Edition), 2013] are usually built around positive economic feedback loops. Initially, a player can generate a resource (like cookies, money, or experience points) through rote clicking on the game interface (hence the moniker ‘Clicker game’): every click produces a guaranteed amount of resources. The player can then invest these resources into game items that then *automatically* click and/or produce more resources instead of the player, which the player can then reinvest into even better items that produce even more resources per time unit, *ad infinitum*. Playing the game therefore often means to wait (or ‘idle’) and let the game play itself, returning occasionally to spend generated resources.

This—now highly successful—game genre originated in satires on so-called ‘progress mechanics’ in role-playing games (Deterding, 2019): by killing monsters and completing tasks, the player’s in-game character can earn experience points or gold which they can then invest in improved in-game statistics (like character strength) or ‘buffs’ (stronger weapons and armour) that make the character more powerful and thus allow the player to more easily overcome given obstacles. Success and advancement in the game thereby become less dependent on the human player improving their ‘real’ skills (such as reading enemy movements or timing responses), and are more a function of time invested into levelling up the ‘virtual skill’ of one’s in-game character (Schell, 2008, p. 151–152).

Idle games take this virtual skill and progress to the logical extreme. Their demonstrable appeal and market success (Pecorella, 2017) directly contradict the notion that gameplay is only engaging and enjoyable under optimal challenge. They also challenge ACE theories in different ways. Effectance theory can easily account for the ever-accelerating streams of cookies, coins, and other resources flowing on the same click as ever-novel forms of effectance feedback. SDT can similarly conceptualise them as positive competence feedback – with the decided wrinkle that this ‘feedback’ continues in the absence of player action, and its production does not require skill. Where, then, is player competence—‘the exercise, expansion, and expression of one’s capacities and talents’ (Ryan and Deci, 2017, p. 86)? Achievement theory arguably struggles most with Idle games. By necessity of its formal calculus, people should have a very low tendency to approach tasks like Idle game play with very high success likelihoods. Succeeding at Idle games is literally a waiting game, not a ‘standard of excellence’ displaying socially desirable properties – if anything, Idle games still draw derision in many gaming communities. To account for Idle games, SDT and achievement motivation scholars need to search for player-devised goals that create some optimal challenge even in Idle game play. And indeed, some Idle game players engage in the economic meta-game of progressing fastest: identifying optimal investment strategies of what in-game auto-clickers to spend on when to achieve maximum income velocity and acceleration. But as far as we know, this is far from the dominant playstyle (Deterding, 2019). As we will argue, PP can account for players not playing the economic meta-game as enjoying faster-than-expected progress.

Far to the other end of the challenge spectrum sit so-called Soulslike games – a subgenre of action role-playing games shaped by the ‘Souls’ series of video games developed by FromSoftware, from the first Dark Souls (Standard Edition) (2011) to the recent Elden Ring (Standard Edition) (2022). Among other things, Soulslike games are characterised by their high difficulty that make frequent and repeated failure and player character death an expectable core part of their play experience. And yet, these games are again highly commercially successful, with a large and devout fan base pouring dozens to hundreds of hours into each title, and studies demonstrating deep player engagement and enjoyment, despite – and because of – their frequent failure (Petralito et al., 2017). This data pattern does not fit achievement motivation theory. While their very high difficulty makes beating the challenges of Soulslike games a prime candidate for a socially desirable standard of excellence (particularly in certain gamer circles), their resultant very low success probability means that players again ought to steer away from them, towards games where the odds of failure and success are exactly even. To ‘rescue’ achievement motivation theory, we need to assume that Soulslike players judge their subjective success odds to be 50%, either because they are very proficient (Soulslike) players, or irrationally overconfident. SDT accounts can point to implicit player-devised goals as sources of competence-satisfying successes. But sustained voluntary engagement in Soulslike games *over other game alternatives* is hard to explain for SDT: if the intrinsic motivation to play arises from competence experiences, then players should no longer want to play after repeated failure, and when given a choice, switch and stick to games with greater frequencies of success. Effectance theory, finally, can explain the appeal of executing nicely animated attacks regardless of repeated player character deaths in enemy encounters. But often-immediate and continued player death creates a comparatively slower rate of effectance feedback and encounter of different enemies, weaponry, etc., which reduces novelty in effectance. In a world of cheap, abundant games, why do not players seeking to maximise novelty in effectance drift to other titles?

### Summary

To explain the appeal of optimal challenges with some uncertain success, current games research chiefly uses ACE theories which argue that we seek and enjoy experiences of *doing well*. Yet on a closer look, these theories struggle to account for the appeal of near-certain success (in Idle games), uncertain success (with optimal challenge), and near-certain failure (in Soulslike games). Achievement motivation theory offers a strong formal explanation for optimal challenge – it maximises the expected utility of success probability times achievement signaling value –, but for that very reason cannot explain Idle and Soulslike games that deviate from this formal optimum. Effectance theory nicely matches the ample ‘juicy’ feedback of Idle games, but mismatches the comparatively sparse and stunted agency feedback of high-difficulty Soulslike games, and offers no direct explanation for why more uncertain success should be more engaging. SDT allows to ‘switch tack’ to find sources of positive feedback on a player’s capacities in Idle games (making strategic investment choices) or Soulslike games (moment-by-moment successes), but is incoherent in its account of optimal challenge. Because it sees intrinsic motivation flowing from positive experiences of *doing well*, it cannot answer why people would not rather drift toward gameplay with the highest success odds.

Having laid out the puzzle of the appeal of uncertain success, likely success, and likely failure in games, we will next introduce core concepts of predictive processing, to then demonstrate how it can account for these puzzles.

## A gentle introduction to predictive processing

Predictive processing (henceforth ‘PP’) is an increasingly influential neurocognitive framework of cognitive processes and how they are materially realised in the human biological system (Hohwy, 2013; Clark, 2015; Nave et al., 2020).^5^ This framework posits that our cognitive architecture revolves around an overarching principle of *prediction error minimisation*. The basic idea is that the human brain constantly generates predictions about sensory observations and their hidden causes in the world and the body, and compares those predictions with actual observations. Mismatches generate *prediction errors*, which are then sought to be reduced, either by correcting our predictions (through passive inference or *perception*), or by making events in the world conform to existing predictions (through active inference or *action*). Importantly, PP terms like prediction, error, expectation, belief, or uncertainty describe mathematically formalised properties of components of its proposed cognitive architecture that operates primarily sub-personally – e.g., as Bayesian probability distributions over alternative beliefs.

In PP, predictions are produced by *generative models* made of the agent’s prior beliefs, i.e., current internal models of the statistical structure of their body and environment, the agent’s own action sequences (called ‘policies’), and how these policies produce state changes. Observations that fit predictions are ignored, whereas *unexpected* observations generate prediction errors. Errors are resolved through interdependent processes of updating of the generative model’s predictions or changing sensory data to fit with the model’s predictions. Both predictions and error-based updating are assumed to flow across a cortical-processing hierarchy that constantly maintains and updates cascading and interdependent predictions which span increasingly longer and more extensive spatial and temporal intervals.

Biological and psychological needs like nourishment or warmth are construed as strong fixed prior expectations of desirable states: observed low blood sugar or body temperature create strong prediction errors, which agents resolve with choosing actions they expect to bring both back to expected baselines (e.g., make and drink a hot chocolate). An agent that regularly succeeds in reducing prediction errors will thus not only succeed in making inferences that best explain the regularities in its sensory states (and improve its generative models): it will also choose actions that tend to satisfy the agent’s needs.

Logically, agents cannot directly determine the course of action that minimises actual prediction errors, as this would require perfect knowledge about future consequences. To optimize action, agents therefore rely on their generative models to estimate which prediction errors – and reductions thereof – to expect given a policy. That is, agents act to reduce *expected prediction error* (e.g., we choose to make hot chocolate because we *expect* this to quickly nourish and warm us). In some influential accounts of PP, *uncertainty* is used to refer to this expected prediction error on multiple levels – from the current state of the world to action selection, future states, the structure of the world, and the structure of our own model of it (Friston et al., 2017). Following this account, uncertainty reduction provides a powerful unifying formal calculus for all different forms of motivation. First, agents aim to maximise extrinsic or *pragmatic value*, that is, reduce the discrepancy between expected desired goal states and observed states, and aim to minimise *risk* in the form of the expected likelihood with which different policies will get them closer to the goal state. Second, agents aim to maximise intrinsic or *epistemic value*, that is, choose actions that promise to reduce *ambiguity* or uncertainty about states of the world. Third, agents aim to maximise *novelty*, that is, choose actions that reduce *ignorance* or uncertainty about how (future) states and actions hang together with (desirable) outcomes. Actual action planning incorporates all these terms to select the action that maximises *overall* expected uncertainty reduction, where different terms can weigh stronger and interact.

Put differently, PP revolves around sub-personal cognitive uncertainty conceptualised as *expected prediction error*. In playing a game, a player wants to reduce uncertainty in the form of (a) pragmatic risk (getting closer to their goal by choosing the actions most likely to get them there), (b) epistemic ambiguity (sampling more information to get a grip on the current game state, especially in games with hidden information), and (c) novelty, exploring the game to discover new entities and actions. Different degrees and changes in salient cognitive uncertainty may then afford different kinds of felt uncertainty and related epistemic emotions—‘aha’ moments, surprise, suspense, etc. External uncertainty (like the randomness of card draws in Blackjack) is something the player would learn to predict better over time to the extent possible. As a player engages with, e.g., the game of Blackjack, their generative models are tuned from observation to (sub-personally) predict the likelihood of certain cards coming or hands winning given the cards played, more and more approximating the remaining irresolvable external uncertainty of the current game state.

### Precision, salience, and attention: Seeing affordances

In PP, uncertainty reduction also drives attention. *Salience*—standing out in perception and drawing attention—in PP is determined by expected information gain or resolution of uncertainty (Parr and Friston, 2018). This has been used to develop an affordance account in PP (Kiverstein et al., 2019): as we orient ourselves in the world, opportunities for action that are salient for attaining our goals or resolving other uncertainty stand out as inviting or soliciting affordances. Attention is further tuned by how much confidence an agent places in the different predictions it makes: the so-called *precision* of predictions (Clark, 2015). Predictions with high precision (high confidence) elicit strong prediction errors if they are violated, whereas prediction errors related to predictions with low precision are typically ignored. The agent will be more surprised and pay more attention—preferentially sample for more observations—when observations fail to match a high-confidence prediction. Similarly, high-precision policies will elicit stronger prediction errors and attention if they turn out to not bring about predicted consequences.

### Affect, mood, and error dynamics: The good feeling of doing better than expected

In optimising for overall expected error reduction, the efficiency of different policies matters. As PP is a dynamic model of ongoing action-perception loops, this efficiency can be captured as temporal dynamics in error rates or *error dynamics*, specifically, changes in the rate of change over time, i.e., acceleration. Thus, an agent is believed to assess how efficiently different action sequences will reduce expected prediction error and pick the most efficient one. If an error reduction rate accelerates compared to a baseline velocity, this corresponds to the agent performing *better than it expected*. Conversely, a deceleration of error reduction corresponds to the agent performing *worse than expected*.

Recently, error dynamics have been used to develop a PP account of emotional experience, particularly affective valence and mood (Joffily and Coricelli, 2013; Van de Cruys, 2017; Kiverstein et al., 2019; Hesp et al., 2021). Valence is commonly used to refer to the felt positive or negative character of our affective experience, which expresses an overall appraisal of the environment as doing well/poorly, helpful/harmful, rewarding/threatening relative to our current state and motivations (Barrett, 2006). Following PP accounts, momentary affective experiences of positive valence are elicited when an agent is reducing error *faster than expected* (i.e., when error reduction accelerates, assuming an expected baseline speed), while negative valence arises under *slower than expected* error reduction (i.e., error reduction decelerates). Mood as a generalized and lasting affective state expresses the agents’ overall expected momentum or direction of error reduction rates: when things repeatedly go worse than expected—error reduction decelerates or even reverses into error increases, we start to form a generalized pessimistic expectation that things will go poorly, which is experienced as negative mood. When things repeatedly go unexpectedly well—error decreases—we form general optimistic expectations, experienced as positive mood. Mood will steer the agent to preferentially choose cautious or optimistic action policies (Kiverstein et al., 2020; Hesp et al., 2021).

### Play, consumable error, and designer environments

A crucial upshot of this sensitivity to and optimisation for efficiency in the form of error dynamics is that predictive agents are not just homeostasis-orientated (seeking stable absence of error), but are also heterostatic or growth-oriented: In a quest for positive valence, they steer toward situations and policies that they expect to improve their error reduction rates relative to past rates, thus growing their active and passive inference capacities. If an action policy then actually reduces error faster than expected, agents will feel good and update their beliefs about the expectable error reduction rate of these actions. Over time, the new observed error reduction rate will inform and become the expected error reduction rate—a ‘hedonic treadmill’ effect where continued progress at the same rate will elicit less positive valence over time. We are still *doing well*, but no longer *better than expected*. And as our confidence in the current action policy increases, so uncertainty about it decreases. Instead of sticking to the current action policy, agents will thus drift to affordances that promise new uncertainty to reduce faster. Paradoxically, this means that agents that care about nothing more than prediction error reduction will search for surprise and error all the time and even sometimes deliberately create it. Uncertainty-reducing agents, in other words, will be intrinsically motivated to engage in exploratory play, and experientially enjoy play if and when the thus-generated uncertainty is then reduced surprisingly quickly (Andersen et al., 2022).

In natural environments, this drive to reduce error at a better-than-expected rate lets predictive agents drift towards niches that are replete with *consumable errors*—that is, situations that agents expect and observe to be neither too complex to manage, nor too predictable and devoid of new information (Andersen et al., 2022; Miller et al., forthcoming). For instance, to most people, a high, straight, and smooth pole in the middle of an empty parking lot offers little consumable error: we expect it to be unlikely that we can climb to the top of it, and there is no new information to gain from the view atop. In contrast, a tree with a rugged bark and many robust branches that slopes gently up and opens an unknown view onto the grounds of a celebrity villa at its top promises much consumable error: it becomes salient as invitingly climbable because we expect that we can climb it, and we expect that the view from the top will reliably and quickly reduce epistemic and novelty uncertainty about what lies beyond. Situations like these hit a ‘sweet spot’ in that they allow agents to encounter significant amounts of prediction error that nevertheless remains ideally and expectably reducible and thus allows agents to do better than what they initially estimated (Kiverstein et al., 2019).

Humans live predominantly in cultural environments or ‘designer environments’ (Clark, 2018, p. 275) that are often purpose-built to maximise enjoyable (and learning-supportive) consumable error. Along these lines, philosophical and empirical aesthetics have become increasingly interested in PP as a promising explanatory framework for the appeal and aesthetic experiences found in visual art, film, music, or literature (see Frascarolli et al., 2021, for a literature review). While it is beyond the scope of this paper, a growing body of evidence and argument supports that media and art are purpose-built to afford consumable error whose build-up and reduction generates aesthetic experiences of suspense, interest, surprise, insight, aha moments, and delight.

## A predictive processing account of the appeal of uncertain success in games

Returning to games, we set out three forms of uncertain success manifest in popular genres: (1) uncertain success of balanced challenges (found, e.g., in multiplayer games with matchmaking), (2) near-certain failure (in Soulslike games), and (3) near-certain success (in Idle games). How does PP account for their appeal?

The answer PP provides is the same as for any other kind of human activity: Humans continually seek to reduce uncertainty or expected prediction error in its various forms (pragmatic, epistemic, novelty-related), and experience positive affect when they do so more efficiently than expected, which leads them to preferentially choose actions that bring such faster-than-expected reduction about. In everyday terms, we seek out *doing well* and seek out and enjoy *doing better than expected* – in attaining goals, understanding the world we are in, and learning how to improve both.

Like other art forms and aesthetic practices, well-designed games are designer environments that afford rich sequences of consumable uncertainty at just the right rates and levels. As multimedia, video games can provide the same range of artificial uncertainties afforded by other art forms: narrative or musical suspense; novelty, complexity, and variety in sound, imagery, plot, characters, or subject matter. But in addition, games afford the particular uncertainties involved in the ‘voluntary attempt to overcome unnecessary obstacles’ (Suits, 2005, p. 43).

In choosing to pursue a particular *goal*—posed by the game or self-devised by the player, players generate ‘unnecessary’ prediction errors which they are then motivated to reduce. Goals in PP are modelled as predicted future sensory observations. These predictions give rise to prediction errors since the goal has not yet been attained: observation tells us that we have not beaten the boss monster or crossed the chasm yet. Once a goal has been formed, the actor needs to infer and pursue the sequence of actions that has the highest probability of leading to the goal state—acting so as to efficiently minimise expected prediction error, or the delta between the goal and what they actually expect and observe to happen next. This basic consumable uncertainty of goal pursuit can become richly laden with additional consumable uncertainties: epistemic ambiguity about where the chasm is narrow enough to cross; quasi-pragmatic uncertainty and risk about what to do (should we jump from the chasm edge or an elevated tree nearby) and whether our jump will succeed; ignorance about the attack patterns and weak spots of the boss monster, or what strategy we could even pursue to beat it. Put differently, many of the various forms of felt uncertainty recognised in games research (Kumari et al., 2019) arise from cognitive uncertainty as understood in PP (i.e., as expected prediction errors). And this cognitive uncertainty in turn emerges around the various forms of external uncertainty entailed in pursuing game goals (Costykian, 2013).

Gameplay differs from other pragmatic goal pursuits in that its designers and players actively lean into amplifying such cognitive uncertainty for the sake of the enjoyment that reducing it provides. Games amplify, but also apportion and sequence their uncertainties so that players can reduce them reliably, and reliably faster than expected. Uncertainty in games *motivates* us to reduce it and holds our attention if we predict that we can reduce it. We *enjoy* games—experience jolts of positive affect—and preferentially engage in them because and when they let us improve the rate at which we reduce their uncertainty. Such improvements will often be accompanied by achieving the pursued goal or winning. Yet what we positively enjoy is not winning or goal attainment itself, but the experience of *improving*, *getting better*, or formally, *accelerating prediction error reduction* relative to our prior expected rate. If we observe that we finish a racing game first after repeatedly finishing last, this sharply reduces error relative to our expected error (we may have expected with high certainty to finish last again). Accelerated error reduction often arises from improved generative models—that is, the player getting better at playing the game. But as power-ups or Idle games demonstrate, accelerations can also stem from game state changes increasing the input/output efficacy of player actions.

Notably, goals, expected error reduction rates, and experienced improvements flow from and occur across all levels in the hierarchy of the generative model: Players may articulate goal states very locally (work out how the merchant mechanic works) or globally (win the *Magic: The Gathering* world championship). Expected error reduction rates may be set by global everyday life experiences (‘I cannot get anything right today’), general expectations about games (‘… but I’m usually quite okay with gaming’), and/or genre- or game-specific expectations (‘… and at least with *this* game I know I will not suck’). Expected error reduction rates will be shaped and continually updated by direct observation (personal play) and received observation (media and social exchange; Iacovides et al., 2015, p. 217). This will attenuate motivation and experienced enjoyment accordingly: players will self-devise goals based on their expectations and be motivated to play as long as they still expect to make progress toward them. They will be frustrated if they expect with high certainty to excel and yet only perform so-so, and delighted if they unexpectedly do well at a game they expected to be hard. Experienced doing better than expected can be similarly local—mastering the button combination and timing in triggering an evasive backflip—or more and more high-level: defeating a monster without taking damage, completing a level without dying, finishing a game on Nightmare mode.

### The puzzle of optimal challenge

How does the PP account of the attractiveness of games we have just outlined explain the appeal of optimal challenges? First, there needs to be *some* perceived-relevant and perceived-reducible uncertainty for a player to be motivated to act. We will not preferentially approach a game challenge we think irresolvably hard because we expect not to be able to reduce the associated prediction errors. Similarly, we will not preferentially approach a game challenge we consider utterly predictable in that we expect with high certainty we will overcome it, as it affords little expected resolvable uncertainty (Andersen et al., 2022). In addition, for a game to be positively enjoyable, there needs to be room for improvement in the player’s rate of prediction error minimisation. In a game that a player has ‘exhausted,’ like *Tic-Tac-Toe* for most adults who spent some time with the game, the player knows with high certainty the optimal strategy for playing, and that they are able to execute it. Thus, there is no inviting prospect of doing better than expected (or reducing ambiguity or novelty) in goal pursuit because there is nothing further to learn, no remaining uncertainty about what to do and whether they can do it, nor will there be any positive experience when playing the game: at every step, our approach to victory (or draw against an equally wise opponent) never exceeds our prediction.

Our attention is drawn to a given game goal (or one that we frame on our own) often because it is perceived to afford the right kind and level of consumable uncertainty: based on past experience, we need to be reasonably confident that we can reduce the presented uncertainty (i.e., that we can find and execute sequences of actions that will attain our goal), and ideally, we expect that we will experience some enjoyable improvement in the course.

Optimal or ‘balanced’ challenges—and initially, the *expectation* of balanced challenges—afford just that. In single-player games, balancing (Schreiber and Romero, 2021) and related design practices like tutorial design (White, 2014) or rational level design (McEntee, 2012) commonly involve crafting a sequence of environments and obstacles that teach and then require mastery new game mechanics or ‘verbs’ in new variations and combinations. In a platformer like Super Mario Bros (Standard Edition) (1985), that may be first teaching and then demanding to jump, then shoot, then jump-and-shoot, then double-jump, then shoot and double-jump, etc. A puzzle game may first introduce the basic puzzle mechanic (connect dots of the same colour with lines), then an extension (you can merge colours, e.g., blue and yellow to get green), etc. This is often accompanied by progression systems where the player’s character increases in virtual capabilities over time: stronger gear, more health, etc. Thus, the player has ideally a constant sense of improvement in both overcoming familiar obstacles faster or easier than before and facing ever-new obstacles with some ever-new uncertainty that, too, gets quickly reduced. If we say players are ‘bored’ by trivial obstacles, in PP terms, this means that players who repeatedly face obstacles for which they have identified high-precision action policies will no longer experience positive affect over doing better than expected (as they now expect to do as well as they do). If we say obstacles are ‘frustratingly hard’, in PP terms, this describes gameplay situations where players repeatedly resolve error less efficiently than expected, evoking negatively valenced affect, until players feel that they can get no ‘grip’ on the situation, that is, they cannot discover an action policy that allows them to improve their error reduction rate, until they lose confidence that they will be able to resolve error at all and quit.

Thus, from a PP perspective, the appeal of uncertain success in optimal challenge is no puzzle at all: A challenge motivates to the precise extent that it affords expectably reducible uncertainty (which moderately difficult game goals do), while enjoyment or positive affect arises from improving or *doing better than expected* at attaining success. Importantly, for PP, enjoyment is maximised not (just) when outcome uncertainty is maximised and then reduced,^6^ but when it allows the player to observe *the starkest improvement in their expected error reduction*.

### The puzzle of idle games

If that is the case, why are Idle games appealing, where success and progress are utterly predictable? In the first order, what is enjoyable and engaging from the perspective of PP is *better-than-expected progress* toward one’s goals, irrespective of whether that progress requires player skill. Progress mechanics like level-ups, new unlocked abilities, new gear can all give us the experience of accelerated error reduction, as we suddenly beat monsters faster, jump further, persuade NPCs that were previously impervious. Think for instance of how a flower power-up in *Super Mario Bros.* allows one to do better than previously expected. In his new state, Mario is newly able to shoot enemies from afar and thus complete the level in a more efficient way. For this reason, picking up a flower and blasting away enemies in *Super Mario Bros.* feels good, at least until one has played the level so many times that expectations have attenuated and the flower pick-up is expected.

The ‘fake progress’ of Idle games is not fake in that it still marks such progress within and against the constraints set by the game world towards the player’s self-set goals, such as discovering the effect of the next upgrade, reaching a new order of magnitude, etc. And this is experienced with positive valence when and because such progress or error reduction accelerates relative to expected rates.

Cookie Clicker (Standard Edition) (2013) is a good example of a game that is designed to give players the experience of continually doing better than expected. Players start clicking a big cookie, where every click generates one cookie as currency. As they reach a certain threshold, new upgrades are unlocked that they can purchase with cookies. These upgrades either automatically generate cookies or add a multiplier to how many cookies each player click generates. Thus, with each purchase, cookie production *accelerates*: the rate of cookies produced per second goes up, and so the player is now doing better than before.

Now one may argue that over time, players will learn to expect not just a steady speed of cookie production, but also regular accelerations with every purchase. This is where the kind of upgrades *Cookie Clicker* offers comes in: while some upgrades are incremental, producing linear accelerations, many upgrades produce compound effects or step changes in the order of magnitude of cookie production speed, accelerating on an exponential curve (Pecorella, 2017). This reliably exceeds expectations—our learned human global expectations for life are linear increases over time (Wagenaar and Timmers, 1979). This, we argue, makes up a basic appeal or sense of getting better in Idle games in addition to that of players improving their actual competencies at the economic meta-game of optimising resource investment choices in Idle games.^7^

One further upshot of the reliable progress structure of Idle games is that one might expect these games to be particularly attractive to players whose life circumstances are highly volatile or frustrating. Such life circumstances set global expectations for error reduction with respect to one’s goals low (Kiverstein et al., 2020). Relative to this irreducible uncertainty in everyday life, Idle games can give players the reliable experience of doing better than expected, thus providing a lift in mood. This aligns with recent arguments and meta-analyses on the recovery potential of ‘easy’ videogames for treating low mood, stress, anxiety, or depression (Pine et al., 2020; Reinecke and Rieger, 2021).

### The puzzle of soulslike games

Where Idle games afford reliably doing better than expected, Soulslike games on the surface can be said to do the opposite: Their mechanics and controls are intentionally not fully explained to players. Many enemies jump from positions or have behaviour patterns that cannot be predicted in advance: a player has to encounter them first (and likely die in the course) to learn them. Most mechanics have minimal error tolerance. Thus, as part of the core gameplay, players will reliably fail and die over and over again in the course of learning the game. How is that any fun?

This question is elegantly dealt with in PP by highlighting the intricate role of *expected* error reduction rates. First, based on prior media coverage or experience, most players will come into Soulslike games expecting repeated failure and slow progress. In PP terms, players expect a very low error reduction rate, and so an actually observed low error reduction rate is not or less frustrating. Again, what matters for motivation and enjoyment in PP is not *doing well per se*, but *expecting* to do well (reduce error) and then *doing better than expected*.

This matches recent empirical work on struggle and failure in video games (Frommel et al., 2021) and Soulslike games in particular (Petralito et al., 2017). Following Frommel et al. (2021), players *expect* ‘temporary failures’ and continue to tackle them as long as they have some ‘belief in success’. Such temporary failure could flip into perceived ‘perpetual failure’ or ‘the continued lack of progress towards players’ goals, which would undermine belief in success until players quit. In fact, players attributed failure and frustration to ‘unsuitable expectations’. This reflects a PP account of continuation motivation as tied to expected consumable error to the dot. Players will stop playing not when they repeatedly fail, but when they stop expecting to make any progress in reducing error. Thus, for players who continue to engage in Soulslike games, PP would predict that difficulty is never such that prediction error levels are completely unmanageable. Soulslike games still provide the – suitably competent and prepared – player with *some* consumable error that allows them to experience improvement.

As for positive affect or enjoyment, Petralito et al. (2017) found that although moments of ‘difficulty & failure’ are the most frequent reported playing Soulslike games, there were also frequent experiences of ‘learning & improvement’ and ‘achievements & victories’. Learning and improvement were most predictive of positive affect, even though they were typically evoked by avatar death, challenging moments and difficulties in general. This makes perfect sense from a PP perspective: what matters for positive affect is not winning, losing, dying or surviving, but *doing better than expected* –improvement, making progress even in or through failure.

So what are sources of improvement in failure? Here the hierarchical structure of generative models in PP comes in: at any moment of gameplay, players can pursue and register incremental improvements at a wide range of different levels, e.g., reading enemy animations, timing moves, discovering a potential new attack strategy, learning a spawn point. As one player puts it: ‘Obviously I died a lot, but every time I learned something new’ (Petralito et al., 2017, p. 1060). This ties in with the fact that reducing uncertainty of any kind is making progress. So even if a player makes no progress in reducing pragmatic uncertainty of beating a difficult boss, they may reduce epistemic or novelty-related uncertainty in learning the game state or trying out and observing the effects of alternative strategies. This is compatible with one player’s description of a difficult boss fight: ‘I learned the right timing to evade his attacks, the right time frame to bring in a few hits myself and when to step back and heal’ (Petralito et al., 2017, p. 1060). This aligns with what Frommel et al. (2021) describe as ‘goal setting as self-challenging’: success and failure is experienced not so much relative to the outwardly observable or predetermined goals set by the game designers, but by the goals players set for themselves—which again can be at any organizational level of gameplay.

Another upshot of the PP model of comparing expected and actual prediction error reduction rates is a logical explanation of the intensity of positive valence reported by players who succeed after continued failure. Through repeated failure, Soulslike games arguably set baseline expectations of small incremental error reduction rates and repeated failure in achieving desired goal states. Against this relatively high-precision expectation of failure, actually getting a win, in other words doing *way* better than expected, can generate an intense feeling of euphoria. As one player reports: “My best experience yet was when I fought the Dancer of the Boreal Valley. It took me a total of 6 h attempting to beat her […] once I beat her, there has been no better feeling of satisfaction than seeing her hit the ground’ (Petralito et al., 2017, p. 5091). Another player reports: ‘The feeling you get after some tries, when you start to think something is just impossible and then you get through a difficult part of the game…. That feeling is indescribable” (Petralito et al., 2017, p. 5091). As Frommel et al. (2021) put it, ‘temporary failure (the struggle) is integral to the experience of success (overcoming the struggle).’ Expressed in PP terms, repeated temporary failure sets low expectations for success while still reducing epistemic and novelty-related uncertainty about how to win (= learning), such that success becomes likelier and when it happens, manifests enjoyable faster-than-expected error reduction.

## Discussion

In this article, we have argued that existing ACE theories struggle to account for the motivational pull and positive experience of uncertain success afforded by optimal challenge in balanced games, near-certain success in Idle games, and near-certain failure in Soulslike games. In contrast, we argued that PP provides a promising explanatory framework for all three. According to PP, humans aim to reduce uncertainty or expected prediction error as efficiently as possible and are therefore sensitive not just to absolute error, but also to changes in the rate of error reduction: positive affect emerges when error reduction accelerates, that is, when we are doing *better than expected*. This core mechanism explains the appeal of uncertain success in games. Trying to overcome a novel game challenge affords uncertainty for the player to reduce, generating jolts of ‘fun’ when this happens *faster than expected*, that is, when the player improves. Positive mood is maintained where the player predicts steady improvements in their error reduction rate. However, learning improves players’ actual and expected error reduction rate for a given challenge. Thus, with learning, uncertainty or expected error over a given challenge goes down, and players get used to the new error reduction rate. Players keep *doing well*, but slow-down in their rate of improvement, until they stop *doing better than expected*. As players aim to maximise the velocity of uncertainty reduction, they will thus preferentially sample new challenges that promise more uncertainty to reduce faster.

### Explaining optimal challenge, idle games, and soulslike games

Optimal challenges are optimal in that they afford not maximal, but maximally *consumable* uncertainty: they concentrate additional artificial uncertainty around the core uncertainty of goal attainment, but in a form that keeps uncertainty increasingly reducible, promising and realizing steady jolts of improvement. PP emphasises that uncertainty reduction continually occurs across all levels of a player’s cognitive hierarchy, paralleled in the different organizational levels of gameplay and player goals—from moment-to-moment, move-by-move to episodes, matches, and live-long improvement.

Idle games similarly afford reliable experiences of faster-than-expected progress *via* upgrades that accelerate the speed of their core resource generation. Specifically, they feature upgrades which repeatedly increase progress on an exponential rather than linear scale—which is the human baseline expectation.

Soulslike games, finally, afford consumable error and sometimes intense positive improvement experiences across different organizational levels of gameplay despite and through failure by modulating player expectations: Players enter the game expecting a low error reduction rate, which reduces felt frustration as *un*expected deceleration of error reduction. Meanwhile, failures reveal information about the game that gradually improves players’ predictive success or ‘grip’ on the game. Players thus keep reducing uncertainty and even *doing better* in small incremental ways, with jolts of intense fun when a challenge is finally overcome: past repeated failure set a very low expected error reduction rate that makes overcoming the challenge positively stand out. Like any other game, Soulslike games stop being enjoyable when expected error reduction velocity is reduced to zero: from repeated failure without any newly revealed information or improved skill, players come to expect that keeping playing will not produce any progress.

### Relation to existing theories

PP sees motivation and enjoyment arising expected prediction error (=uncertainty) reduction rates. This aligns with (and provides an explanatory framework for) increasing bodies of empirical research identifying the importance of expected versus actual success or difficulty in game engagement (Iacovides et al., 2015; Lomas et al., 2017; Denisova and Cairns, 2019; Frommel et al., 2021). People are *motivated* to start, continue, or stop playing based on expectations of being able to progress—reduce error. *Enjoyment* arises from error dynamics, when the delta between expected and observed error is reduced a rate that is greater (e.g., faster) than expected. This implies that it is not absolute rates of success, positive feedback, achievement, etc. that matter for enjoyment (*doing well*), but improvement or learning progress relative to expectations (*doing better than expected*). Whereas other theories argue that positive experiences motivate play, PP argues that expected error reduction motivates play, while changes in expectation/observation deltas give rise to positive (or negative) experience and update expectations.

This error dynamics model marks an important difference to ACE theories that can answer to some of their shortcomings, such as the incoherence in SDT’s optimal challenge account. SDT starts from the plausible intuition that if intrinsic motivation is an activity-inherent enjoyment that fuels growth, then situations that are most growth-inducing—presumably, moderately difficult tasks—should be the most enjoyable. The incoherence stems from then conceptualising the underlying motive and enjoyable experience, competence need satisfaction, as a sense of doing well, which is logically maximised under easy tasks. Exchange this with a dynamic, comparative sense of doing better, and logically, enjoyment is maximised under tasks with the starkest improvements in reducing predicted errors. An error dynamics model is *directly* sensitive to growth or learning (the more we improve, the better we feel).

But as we noted, it does not immediately distinguish between improved expected error reductions due to player competency growth and those evoked by game design (like power-ups, juicy feedback, or exponential progress curves).

PP’s error dynamics model also explains White’s (1959, p. 322) claim that sustained effectance experiences require continued novel ‘difference-in-sameness.’ For PP, effectance can be construed as the felt exhaust of ‘low-level’ cognitive uncertainty reduction over action policies: e.g., I shoot and hit an enemy as I predicted. Effectance as a *salient, positively valenced* experience depends on better-than-expected uncertainty reduction: I predict to shoot and hit, and the shot hits an unexpected gas tank on their back, producing a massive explosion that kills multiple enemies at once. Such juicy feedback can be positively experienced because it exceeds baseline life expectations about everyday agency (where outputs are proportionate with inputs). This then over time gets attenuated by observations updating expectations to game-specific, genre-specific, and game-general baselines: we learn to expect juicy feedback with high certainty, such that *non*-juicy feedback stands out negatively, and continued positive effectance experience requires novel accelerations in uncertainty reduction.

### Relation to practitioner models

In parallel to and sometimes inspired by academic models like ACE theories, designers have been developing their own theories of gaming motivation and enjoyment, where overcoming optimal challenges again often takes centre stage (see Bateman, 2015, for a critical analysis). Maybe the most influential among these is Koster’s (2005) book-length *A Theory of Fun for Game Design.* Along several lines, his account aligns well with the PP model we propose.

Manifestly inspired by schema-theoretical approaches in cognitive psychology, Koster proposes that perception, cognition, and action revolve around *pattern recognition*: Learning for Koster means identifying and forming internal representations of recurring patterns in sensory data (Koster, 2005, p. 21). As learning is useful for survival, our cognitive systems have evolved to intrinsically reward it with pleasurable experience or fun: ‘Fun, as I define it, is the feedback the brain gives us when we are absorbing patterns for learning purposes’ (Koster, 2005, p. 96). Games lend themselves particularly to evoke this ‘pleasurable learning experience’ (Koster, 2005, p. 44) because they are designed to afford low-risk repeated exposure to sense data that is custom-designed for faster-than-usual pattern learning: ‘Games are […] concentrated chunks ready for our brains to chew on. Since they are abstracted and iconic, they are readily absorbed. Since they are formal systems, they exclude distracting extra details. Usually, our brains have to do hard work to turn messy reality into something as clear as a game is’ (Koster, 2005, p. 36). This optimal design for continuous, fast, pleasurable learning also requires striking ‘just-right’ levels of signal-to-noise, of ‘pacing of the unveiling of variations in the pattern’, and of pacing new patterns to learn (Koster, 2005, p. 44). This is where optimal challenge comes in: ‘Real fun comes from challenges that are always at the margin of our ability’ (Koster, 2005, p. 97).

PP and pattern recognition mark different research traditions in cognitive science—particularly, pattern recognition assumes a more traditional passive, ‘bottom-up’ model of perception and action than the active inference process proposed in PP. But many main principles are shared: Both Koster and PP agree that jolts of positive affect or fun arise *not* when we *do well* (as ACE theories would have it), but when we *get better* or learn something new: ‘Fun is primarily about practicing and learning, not about exercising mastery’ (Koster, 2005, p. 96). Balanced or optimal challenge is not a state of maximal success, but maximal *velocity of progress*, afforded by consumable error: ‘As we succeed in mastering patterns thrown at us, the brain gives us little jolts of pleasure. But if the flow of new patterns slows, then we will not get the jolts and we’ll start to feel boredom. If the flow of new patterns increases beyond our ability to resolve them, we will not get the jolts either because we are not making progress’ (Koster, 2005, p. 98). What Koster describes as information and puzzles presented in simplified form and just-right pacing aligns neatly the PP notion of consumable error and changes in error reduction velocity.

### Implications and outlook

We have argued that PP offers a coherent explanatory model of engagement and enjoyment from uncertain success. Beyond that, we think that PP holds several further opportunities for games research. First, while we here expressly avoided mathematical formalisms to make PP accessible to new readers, PP is fundamentally a (Bayesian) formal model, with fully specified mathematical formulas and computational implementations underpinning verbal descriptions. One refrain of the current psychological reform movement is that most psychological theories – present ACE theories arguably included – exist only as ambiguous verbal claims that make falsification near-impossible (van Rooij and Baggio, 2021). Formal mathematical modelling of theories is a precondition for their severe testing and affords attractive new forms of computational social science research for doing so, such as computational cognitive modelling and simulation, comparing modelling and simulation results with observed human data.

Second, PP’s formal models also open a wide range of practical implementations in digital games. A computational model of motivationally and experientially optimal consumable uncertainty and uncertainty reduction rates could for example be used for automated playtesting (Politowski et al., 2022), experience-driven procedural content generation (Yannakakis and Togelius, 2011), dynamic difficulty adjustment (Zohaib, 2018), or adaptive AI NPCs (Merrick, 2016).

We hasten to add that PP is far from the only formal model of (intrinsic) motivation and positive affect (see Oudeyer and Kaplan, 2009; Oudeyer, 2018, for reviews). In recent games research, Guckelsberger (2020) has proposed and developed empowerment maximization as a compelling alternative computational intrinsic motivation model for video games. In the classification of Oudeyer and Kaplan (2009), both PP and empowerment maximization can be formally characterised as *learning progress* models, and we gladly concede that most such learning progress models offer comparably coherent explanatory accounts of uncertain success. The exciting thing is that by virtue of formal modelling, we have new means at our disposal to actually test these and other different models. Comparative testing can then show which actually tracks human data better than other approaches – and/or actually produces more engaging gameplay.

Finally, this paper intentionally focused on one external uncertainty source—uncertain success. We are optimistic that PP’s model of cognitive uncertainty as expected prediction error may subsume the full range of forms of engaging uncertainty found in games (Costykian, 2013). Current explanations for the pull of these games chiefly point to curiosity not ACE as underlying motives (Kumari et al., 2019). Yet as noted throughout, for PP, pragmatic risk, epistemic ambiguity, and novelty are all forms of uncertainty (expected error) our cognitive system aims to reduce overall in the same mechanism. Thus, PP could also form the starting point for reuniting two strands of psychological intrinsic motivation research that split off in the second half of the 20th century (Oudeyer and Kaplan, 2009): competence models that today dominate games research and other domains, and information-theoretical curiosity models prevalent in empirical aesthetics, which as we noted are increasingly embracing PP. Both may turn out to be fuelled by the same principle: mastering uncertainty.

## Data availability statement

The original contributions presented in the study are included in the article/supplementary material, further inquiries can be directed to the corresponding author.

## Author contributions

SD, MA, JK, and MM: conceptualization, writing-original draft preparation, and writing-reviewing and editing. All authors contributed to the article and approved the submitted version.

## Funding

This work was supported by the EPSRC Centre for Doctoral Training in Intelligent Games and Game Intelligence (IGGI) [EP/S022325/1], the Digital Creativity Labs jointly funded by EPSRC/AHRC/Innovate UK under grant no. EP/M023265/1 (SD), the Lego Foundation (MA), the ERC Starting Grant 679190 (EU Horizon 2020; JK), and the Netherlands Organisation for Scientific Research (NWO; JK).

## Conflict of interest

The authors declare that the research was conducted in the absence of any commercial or financial relationships that could be construed as a potential conflict of interest.

## Publisher’s note

All claims expressed in this article are solely those of the authors and do not necessarily represent those of their affiliated organizations, or those of the publisher, the editors and the reviewers. Any product that may be evaluated in this article, or claim that may be made by its manufacturer, is not guaranteed or endorsed by the publisher.

## Footnotes

^1^This question of uncertain success can be read as an inverse formulation of Juul’s (2013, p. 2) “paradox of failure”: “1. We generally avoid failure. 2. We experience failure when playing games. 3. We seek out games, although we will experience something that we normally avoid.”

^2^Klimmt (2006, p. 91–92) similarly evokes curiosity to explain why players, in the absence of goals or action necessities imposed on them by the game, would actively choose to explore the game’s action and goal space. Once a player chooses a course of action, succeeding at it will then generate competence experiences.

^3^While this definition encompasses both experienced effectance *and* its antecedents (“opportunities and supports”), SDT’s default operationalization in the Intrinsic Motivation Inventory and similar scale only captures experienced effectance, with items like “I think I am pretty good at this activity” (CSDT, 2022).

^4^Atkinson’s full model mirrors the Tendency to Approach Success (*Ts*) with a Tendency to Avoid Failure (*Taf*), with identical terms in reverse: a Motive to avoid Failure (*Maf*), Probability of Failure (*Pf = 1–Ps*) and Incentive value of Failure (*If = 1*–*Pf*). Thus, the overall Tendency to approach a task *Ta = Ts*–*Tf* = (*Ms* × *Ps* × *Is*)–(*Maf* × *Pf* × *If*). The optimal challenge upshot remains that regardless of *Ms* and *Maf* values, overall *Ta* is highest when *Ps*/*Pf* = 0.5.

^5^To introduce PP to a diverse games research audience, we here explicitly avoid mathematical formalisms. Interested readers are directed to the recent introduction and synthesis by Parr et al. (2022).

^6^Of course, taking and observing actions whose outcomes have a high external uncertainty (like a coin flip) *also* very sharply reduces epistemic uncertainty, which adds to the players’ overall uncertainty reduction. We bracket this dimension for future discussion.

^7^We also recognise that the motivational pull of Idle games has been explained with other, non-ACE motives as well, particularly curiosity about new content and story beats being revealed over time (Cutting et al., 2019; Deterding, 2019). While this is beyond the scope of this article, PP elegantly incorporates curiosity as agents optimising *epistemic* and *novelty* uncertainty reduction (Friston et al., 2017; Clark, 2018).
